# Research on Legal Constraints of Individual Environmental Data Rights and Interests in Big Data Environment

**DOI:** 10.1155/2022/4493267

**Published:** 2022-07-11

**Authors:** Yineng Xiao

**Affiliations:** School of Health Humanities, Peking University, Beijing 100191, China

## Abstract

Due to the practical needs, the lack of legal protection, and the lack of attention to these three factors under the existing legal framework of personality rights, these factors together determine the necessity of the establishment of personal information rights. As an emerging right of scientific and technological progress and big data application, how to define the right ownership, right object, and right content of personal information right in theory? Firstly, starting from the theory, this article summarizes the opinions and controversies of the academic circles on the relevant issues and tries to expound its own understanding and views on the basis of comprehensive evaluation. Combined with the introduction to the relevant cases, on the basis of theoretical research, I tried to analyze how to determine the constituent elements of the legal relationship of personal information right in judicial practice, so as to make the theoretical research and judicial practice closely combined. In addition, this article also lists and analyzes the legislative status quo of personal information right protection in twelve countries and regions and expounds three main issues in the legal relationship of personal information right under the background of big data from two aspects of theory and practice: (1) the definition of the scope of personal information; (2) subject identification under the application of network data; (3) a new understanding of the content of personal information right. The conclusion of this article has certain practical significance.

## 1. Research Status

With the development of information economy, data have become the core factor of production in the era of digital economy, integrating into the process of creating economic value and continuously reconstructing economic and social forms and personal life. However, data opening also brings pressure to information security, and the massive collection and use of personal information has aroused people's concern.

Since the application of computer processing and storage of personal information, the Western society began to pay attention to the protection of personal information [1]. In the Common law system represented by the United States, the legislative protection of personal information emphasizes human freedom, and the protection of personal information is based on the right to privacy. The academic circle also studies personal information for the protection of privacy. The protection of personal information mentioned in many research literatures is essentially the protection of privacy interests reflected by personal information itself. In the study of privacy, Samuel Warren and Louis Brandeis published on Privacy in 1890 [2], which gave a simple definition of privacy, that is everyone has the right to be left alone. The publication of the paper had a profound impact on subsequent privacy legislation in the United States. In addition, various scholars have proposed different types of privacy in subsequent studies. Prosser's 1960 article on Privacy divides the right to privacy into four types, which are recognized by most US state statutes. Daniel J. Solove divides the right of privacy into six types, including personal information self-determination. In the process of the development of the later privacy theory, Whalen v. Roe in 1977 formally established that the information privacy right mentioned by scholars in the 1960s was protected by the Constitution. However, due to the development of information technology in the era of big data, people's concept of privacy has changed, and personal information that is traditionally considered private is shared on social media. Omer Tene and Jules Polonetsky conclude that technology is driving changes in social perceptions of privacy. Sun Microsystems CEO Scott McNealy predicted [3], “You'll have no privacy. Forget about privacy.” However, some scholars have raised objections, saying that privacy will not disappear and stressing the protection of personal information. In contrast, the Recent General Data Protection Regulation of the European Union has strengthened the protection of personal information, and some scholars in the United States have called for drawing lessons from the LEGISLATION of the European Union to formulate a special privacy protection law [4]. Some scholars have also expressed their views on the data portraits stipulated in the REGULATIONS issued by the European Union [5] and proposed that accurate user portraits can realize low-cost and large-scale tracking. In general, the European Union and the United States have established different legislative models, and scholars in various countries have combined their own personal information protection models with practice to provide a theoretical basis for legislation.

## 2. Legislative Status of the Protection of Personal Information Right

Table 1 shows the legislative status of the protection of personal information right in several major countries and regions.

Due to the popularity of Internet technologies and applications, personal information is collected, stored, mined, and processed on a large scale, which is necessary for business and social management activities, so countries regulate personal information protection through legislation, in which the European Union and the United States appear as representatives. It reflects two different modes of legislative protection respectively. The European Union mainly protects personal information through uniform legislation. In response to large-scale information collection and utilization in the context of big data, continental European countries took the lead in trying to initiate special legislation, with Germany as the most typical. In 1977, the Federal Personal Data Protection Law promulgated by the German Federal Parliament came into effect, which for the first time systematically and centrally protects personal information and standardizes the collection and use of personal information. The 1995 data protection directive for personal information protection legislation system is the European Union [6]. The most basic provisions of the Act are the right to personal information, as well as the obligations of those who collect or process personal information. It plays a very important guiding role in the protection of personal information in EU countries. In 2012, the EU adopted the General Data Protection Regulation (GDPR) [7], which was revised twice in 2014 and 2016. The latest version came into force on May 25, 2018. Compared with its predecessor, the Eu Data Protection Directive, which was adopted in 1995, GDPR is directly applicable to EU member states, without the need for member states to translate it into national law. The regulation aims to restrict Internet and big data enterprises' processing of personal general information and sensitive information, so as to protect the rights of information subjects [8]. Its application is not limited to the territory of the EU, and the application outside the EU includes two situations: one is to provide goods or services to data subjects in the EU, whether they pay or not; and the second is to monitor the behavior of data subjects in the EU. This means that companies around the world are likely to be subject to the GDPR, which has been described by some media as “the most stringent information protection law in history.” To date, GDPR is the most comprehensive legal standard for the protection of personal information (or personal data) in the international community. It sets a new flag for the international information protection movement and has important reference significance. The United States is the first country in the world to put forward and protect privacy right through laws and regulations and has formed a relatively complete legal protection system for privacy right in China. Therefore, the United States adopts the form of accessory protection of privacy—the protection of privacy is the protection of personal information. To be specific, the protection of personal information in the United States is scattered in all walks of life. Associations of all walks of life and their regulatory departments formulate standards and applicable rules for the protection of personal information in their respective fields. There is no unified personal information protection law. For the public, the Privacy Law of 1974, based on the protection of privacy rights, standardizes and restricts the federal government's behavior of collecting, storing, transmitting, and processing citizens' information through the theory of privacy rights, so as to prevent the federal government from infringing on citizens' information. Facing the market, the United States emphasizes economic liberalization, opposes monopoly, and encourages competition. Therefore, the United States pays special attention to industry self-discipline on the basis of free competition. It adopts a decentralized legislation model for various industries and makes “personalized legislation” for problems arising from the collection and use of personal information in various industries. For example, the Electronic Communications Privacy Law of 1986 and the Children's Online Privacy Protection Law of 1998 [9]. To sum up, the United States adopts a comprehensive protection model of “unified privacy protection + industry self-discipline” for personal information protection, in which industry self-discipline is the dominant. It is worth noting that in 1977, the Supreme Court of the United States first analyzed the right to privacy in Whalen v. Roe, which mentioned the concept of informational right to privacy. This case was the first judgment on the collection of personal information in the United States. Although it did not formally establish the right to information privacy at the legislative level, it indirectly acknowledged its existence, which greatly promoted the development of privacy theory.

Scholars' discussion on personal information right has experienced a transition from privacy to personal information right. Scholars Samuel Warren and Louis Brandeis for the first time published their views in American public journals, believing that privacy is the right of individuals to freely enjoy the privacy and tranquility of their personal life that is exclusive of interference and intrusion. Right to be alone is emphasized [10]. Other scholars have linked the right to privacy to aspects of an “intimate” or “sensitive” person's life, defining the right to privacy as “a state of control over intimate areas of decision-making, including decisions about intimate access, intimate information, and intimate behavior.” From the right to privacy to the right to personal information. With the continuous development of the information society, the application of Internet technology has caused a huge impact on human life [11]. Scholars gradually realize that in modern society, more positive factors should be injected into the right to privacy and the right holder should be given the right to actively protect his personal privacy. After the promulgation of the Privacy Law of the United States in 1974, scholars began to attach importance to the ability of information itself to control its information and put it into the connotation of privacy. Scholars Daniel Solove and Paul Schwartz believe that the protection of privacy is the active control and domination of information subjects over their own information. Alan Westin's definition of privacy takes information control as the core and believes that privacy means that the subject of right has the right to independently decide when, how, and to what extent the information related to himself will be transmitted to others [12]. Scholar Charles Fried believes that the mode of privacy protection should not follow the passive form of the past. On the contrary, with the development of society, people begin to perceive that their personal information should be controlled by themselves [13]. Katrin Schatz Byford, a scholar, defined privacy as “the right to control the dissemination of information about oneself” [14] from a positive perspective.

With the continuous development and in-depth study of these theories, the connotation of privacy gradually began to change, so the concept of “personal information right,” which emphasizes information control, emerged at the right moment [15]. The definition of personal information right. In the case of German census in 1983 [6], the court referred to the right of personal information as the “right of information self-determination,” which mainly means that the subject of information, that is the person to whom the information is directed, controls his or her own information in accordance with the law and decides the flow and use of information according to his or her own will. Therefore, the definition of personal information is particularly critical. According to scholars James B. Rule and Graham Greenleaf, personal information refers to the information that can be directly connected with the identity of a specific individual, or can point to a specific individual in combination with other information. Therefore, identification is the key point to judge personal information. In addition, some scholars believe that only by relying on certain media and being recorded can personal information be called personal information [16]. This is also the second key to personal information judgment, which is treatable. On the relationship between personal information right and privacy right [17], scholars generally agree that the protection of privacy or the protection of personal information right reflects the individual's independent decision on his or her life and reflects the individual's personal dignity and freedom. Whiteman, an American scholar, believes that privacy is the core of maintaining individual dignity and personal freedom. As far as personal information is concerned, people pay more and more attention to it not only because of its gradually prominent property value, but also because of its embodiment of personal dignity and personal freedom [18]. The right to personal information is also known as the “right to information self-determination,” and its connotation also includes the protection of individual personality interests [19]. To protect the personal information of information subjects from technical processing, its core value also lies in the protection of the personal dignity and personal freedom of information subjects [20].

## 3. Constituent Elements of Legal Relationship of Personal Information Right in the Context of Big Data

### 3.1. Scope of Personal Information

As mentioned above, the object of personal information right is personal information. As a new legal concept, different countries have different understandings of personal information, which can be reflected in the appellation of legislation related to personal information in different countries. Some countries call it “personal data,” such as Germany's Federal Data Protection Law; some countries called “personal privacy,” such as Australia's privacy Act. Therefore, before studying the scope of its protection, this article believes that it is necessary to clarify the relationship between personal information and personal data, personal data and personal privacy, and have a clear understanding of the distinction between each other.

#### 3.1.1. Distinction between Personal Information and Related Concepts

Both personal data and private data come from the English word “personal data,” which has different titles due to different translations. There is no substantial difference between them, but both are related to personal identification. Generally speaking, personal information is equivalent to personal information, refers to all information related to the individual, and personal information is only a kind of external presentation of personal information. Similarly, if personal information is stored on a computer or on the Internet, it becomes personal data. Although there is a view that private data or personal data is more focused on the form of information carrier and external performance, personal information is expressed by the information content itself, and the information interaction between the information subject and the content reflects the information between the information subject and the perception subject, which is more inclusive and stable. However, this study believes that the core of personal information, personal data and personal data is the corresponding content of information, rather than what form of information is presented. Therefore, from this point of view, personal data and personal data are no different. In addition, some people believe that the word “data” comes from the English word “data,” which itself is a plural noun. Therefore, data emphasizes the collection for a certain purpose. Then the so-called data (data) is formed by summarizing and recording one piece of information within a certain range. In other words, data is a collective form of information, but there is no essential difference between data (data) and personal information in terms of its core meaning, that is content. Therefore, there is not much discussion on the distinction between the three in academic circles, and the three are often mixed in the legislation of various countries. Compared with personal data and personal data, the legal title of personal information is more humanistic. Therefore, in today's information society, most countries also take personal information as the conceptual basis of their legislation. At present, the academic circles are discussing the relationship between personal information and personal privacy. From the point of view of right status, personal privacy is the form of personal information that the information itself does not want to be disclosed to the outside world in daily life.

There is no limit to states, they can be public or private. In addition, in the context of today's big data, the storage of information has far exceeded the past, and the generation of big data makes the content of personal information complex and diverse. Privacy (especially private information) is only a part of personal information. In this regard, scholars represented by Professor Wang Liming believe that compared with personal privacy, the scope of personal information is significantly wider. At the same time, there is a certain connection between personal privacy and personal information: some personal information, such as mobile phone number and ID number, belong to privacy, but some personal information, such as name and gender, do not belong to privacy. Scholars represented by Professor Zhang Xinbao believe that there is a cross-relationship between personal information, which is not only a sensitive part closely related to personal life but also a category of privacy. However, with the need of social interaction, personal information such as name and contact information is more mobile, so it is no longer classified as privacy. As for the relationship between personal information and personal privacy, scholars mostly discuss about the scope of the two, or the coverage of the object, and there are mainly two viewpoints: the distinction theory and the crossover theory. In the process of literature reading, this article found a new perspective to distinguish and compare personal information and personal privacy, which deserves attention.

Firstly, the connotation of the two is analyzed: Compared with the concept of “personal information,” as the object of privacy, personal privacy means that private life is not disturbed, and private information confidentiality is not illegally collected and disclosed. It can be seen from its expression that personal privacy emphasizes the undisturbed state of a person's private life. It cannot refer to a specific matter and is an abstract concept, while personal information is a specific concept and refers to the information that can directly or indirectly refer to a specific individual. Secondly, there are great differences in value judgment between the two, so it is inappropriate to compare them at the same level. To be specific, personal privacy is the judgment of others on the degree of intrusion into the party's private domain. Due to the need of social communication, each person's private life more or less will be open to others, the private sector is invaded by others, which means that everyone with a certain tolerance obligation; however, the obligation of tolerance is not unlimited. If the degree of intrusion of others on the subject of information is too deep and serious, it infringes on the privacy of the obligee. Therefore, personal privacy is result-oriented and judged by the consequences caused by the violation. Personal information refers to the information that can identify or point to a specific individual and is judged by the identification and directivity of the information itself. In terms of privacy, we can state that a message is personal, but if the context mentions privacy, we cannot determine whether the message belongs to personal privacy, since privacy issues involve value judgments, need combined with specific facts, the influence of the parties, their subjective feelings, and etc., of comprehensive judgment, and personally identifiable information is a question of fact judgment. To sum up, in view of the difference in value judgment and definition between personal information and personal privacy, the two should be clearly distinguished and should not be confused.

#### 3.1.2. Division of Personal Information

Personal information can be divided into sensitive personal information and nonsensitive personal information based on sensitivity [21]. Sensitive personal information, as its name implies, refers to information that directly involves sensitive areas of an individual's private life. According to China's Personal Information Security Regulations, which took effect in May 2018, sensitive personal information refers to personal information that will cause great physical and mental damage or property loss once disclosed or improperly used. EU went into effect in 2018 during the same month the general data protection ordinance, which is about “sensitive personal data” regulation: disclosure of racial or ethnic, political opinions, religious or philosophical beliefs, or trade union members of personal data or can be used to identify specific personal biometric data, such as fingerprints, genetic information, etc. By contrast, nonsensitive personal information refers to information that does not directly involve sensitive areas of a person's private life. According to the Swedish Personal Data Law, nonsensitive personal data/information refers to information that clearly does not pose a great threat to the privacy of the information itself. As mentioned earlier, identifiability is a key factor in determining personal information. Therefore, based on identifiability, personal information can be divided into direct personal information and indirect personal information. Direct personal information refers to the information that itself can be directly associated with a specific individual, that is the information that identifies the information itself. It can be seen that direct personal information has a strong personal directivity, which directly and uniquely corresponds to the information itself. Common direct personal information includes genetic information, fingerprint information, ID number, etc. Indirect personal information refers to the information that itself does not directly point to a particular individual, but after the multiple correlation analysis of information can point to specific personal information, such as name, interests, skills, and talents, and job information such as financial status must be associated with their names, work units, and other information to identify information points to themselves. Under normal circumstances, courts generally protect direct personal information as personal privacy, while there are great controversies in judicial practice regarding the protection of indirect personal information, which will be discussed in detail in the next section.

#### 3.1.3. Determination of Personal Information in Judicial Practice

In China's judicial practice, personal information is mainly protected under the existing framework of privacy right. According to the mentioned in this article, the personal information of infringement cases, courts can be found in that one kind of personal information is protected, more to whether it involves the privacy interests as the judgment standard, the dispute focus on personal information can judge and privacy interests identification measures, such as personal privacy information comprehensive recognition. Specifically, when hearing cases related to personal information, the court will categorize personal information according to the degree of sensitivity. The specific division has been discussed in the previous section and will not be repeated. As sensitive personal information is closely related to the personal dignity and personal freedom of the information itself, the public can generally know that the information itself has strong personal dependence on such information and is reluctant to disclose it to others. Under normal circumstances, sensitive personal information is not allowed to be freely disseminated to the outside world without the permission of the person. Therefore, the court will identify the infringement of such information as privacy infringement, and there will not be much controversy in general. The most controversial cases are those involving general personal information (i.e., nonsensitive personal information) such as names, telephone numbers, addresses, and workplaces. Due to the need of social communication, information such as name and work unit has a high degree of openness, and most people will define it as personal general information. Therefore, whether such information is protected by law needs to be analyzed in specific cases. In tandem with the arrival of big data, new technologies are continuously emerging, among them the construction of a cloud platform and distributed computing provides a basis of big data storage security; artificial intelligence for large data intelligent analysis, mining, and boosting the role of the application of ascension and the application of sensors in the IoT allow for increased access to data. The so-called personal information refers to all kinds of information that can directly or indirectly identify natural persons. It refers to the name, date of birth, ID number, fingerprint, marriage, occupation, marriage, health, property, social relationship, and associated information of natural persons. Any information that can uniquely determine the attribute information of an individual is called personal information. “Personal information” refers to personal information that is private, confidential, hidden, and not intended to be made public. Privacy is a subset of personal information, as shown in Figure 1.

### 3.2. Subject Identification under Network Data Application

#### 3.2.1. Whether Legal Person (or Other Social Organization) Is the Subject of Personal Information Right

Information protection of legal persons (or other social organizations). Legal person (or other social organization) is a legal subject, because of the need to participate in social production and business activities is endowed with rights and capabilities, enjoys legal rights, and bears legal responsibilities. It is true that legal persons (or other social organizations) also produce a large amount of information during their existence, which is more or less related to the vital interests of legal persons and the purpose of their establishment. However, just as there are essential differences between natural persons and legal persons (or other social organizations), there are still partial differences in the information directed towards them: information protection for natural persons is aimed at maintaining personal dignity and freedom, while information protection for legal persons (or other social organizations) is centered on their economic interests. Due to their differences in value orientation and legislative purpose, the established system itself will be different and cannot be adjusted through the same law. Therefore, in the relevant legislation of various countries, the vast majority of countries adopt separate legislation, that is, the information protection of legal persons is separated from the personal information protection law and protected in separate legal norms. For example, The Federal Data Protection Law of Germany does not adjust the data protection relationship related to legal persons, but there are provisions to protect legal persons' information in the Communication Law and the Data Protection Regulations of the Communication Service Industry. In addition, in Chin's legal system, the “personal information” of legal persons, namely trade secrets, can be infringed with the help of anti-unfair competition law, and a special trade secret law may be issued in the future to protect it. Therefore, the subject of personal information right discussed in this article is only limited to natural persons, excluding legal persons and other social organizations. Of course, I do not exclude the possibility and necessity of incorporating legal persons' information into the personal information protection system in the future with the development of society.

#### 3.2.2. Whether the Information Collector Has the Right to Personal Information

When it comes to the application of big data in real life, a large amount of personal information is in the hands of commercial subjects and public authorities. Then do these information collectors have the right to personal information? I believe that the answer is no. The subject of personal information right is still the natural person who produces the original information, that is, the person to whom the information is directed, not the collector of the information. In today's Internet era, all personal information have high liquidity, people's personal information will not be in the form of express or implied government departments or commercial organizations to collect, information gatherer is not the subject of right of personal information at this time, because they only shall have the right to the information that I hereby authorize the limited content, information will be collected in a particular way for a particular purpose. Unlike the information itself, it does not enjoy the complete power to control and dominate its own information, such as the right to deal with inquiries, the right to raise objections, the right to delete requests, etc. Therefore, in the context of big data, the right to personal information only belongs to the information producer (i.e., the person to whom the information is directed), rather than other information collectors or information users.

#### 3.2.3. Whether Information Subjects Are Protected in a Virtual Network Environment

In the network environment, most people publish their information under virtual names, but the information subject in reality has the right to personal information. They just virtualize their real personal information through the network, but the value of their personal information is not diminished, and it still reflects the personal interests of the real information subject. Therefore, the subject of personal information right in the virtual network environment is the real natural person corresponding to the information, rather than the virtual name subject in the virtual network environment. However, due to the virtuality and complexity of cyberspace, it is necessary to determine whether the personal information of the real subject under the virtual name in the network environment is protected by law in judicial practice. With the popularization and application of the Internet, the protection of personal information in the virtual network environment has gradually been concerned. The review process of the newly published Civil Code on Personality Rights (Second Review draft) in April 2019. Some members suggested adding provisions on the virtual identity of civil subjects in order to solve disputes over personal information infringement in the online world. I think that this proposal has its rationality, but how to stipulate it and its legislative effect still needs further discussion and research.

### 3.3. A New Interpretation of the Content of Personal Information Right

As for the content of the right of personal information, it is generally believed that the right of personal information should be reflected in the ability of the information itself to decide and actively control its own information. In terms of the content of the right of personal information, some scholars think that the right of personal information should include the right of information self-determination, the right of information management, the right of permission to use, the right of prohibition to use, and the right to profit. In addition, some scholars believe that information subjects' control over their personal information can be reflected in the following aspects: The person has the right to independently decide whether and how his/her information will be collected and utilized, request others to keep his/her personal information confidential, check the status of his/her personal information when it is collected and processed by others, request to modify or delete his/her wrong information, and request others to pay for the use of personal information. Previous scholars have discussed the interpretation of the right content in terms of controlling and dominating the information itself, but this type of control and dominance is not realistic when considering how to end a number of processing behavior, such as possession, use, open, transfer and analysis, modify, delete, etc. Therefore, I want to interpret the content of personal information right from a new angle. As mentioned above, under the background of big data, personal information right is a new type of right with both personality attributes and property attributes, and personality attributes play a dominant role. In this sense, the right content of personal information right can be divided into personal information personality right and property interest from the perspective of law and economics, so as to reflect the independent value of personality and property use value of personal information, respectively. Specifically, the other benefits of personal information are mainly for the information itself to obtain certain economic benefits, or for a social evaluation or service. The right of personality aims to maintain the integrity and correctness of personal information and personal information in the process of free circulation. The external image of personal information is made to become a kind of real information. Specifically, according to the different stages of information circulation, personality interests include the right of informed consent in information collection, the right of inquiry in information processing, and a series of intervening rights to object to the processing activities of information controllers.

#### 3.3.1. Personal Right of Personal Information

Personal information personality right refers to the integrity and correctness of information in the process of free circulation, so as to realize the value of personal dignity of information. Compared with the passive defense mode of privacy of personal information in the past, personal information personality right in the context of big data emphasizes the active control and domination of the subject of personal information. According to the different stages of information circulation, this control and domination can be further divided into two stages: The first is the stage of information collection, that is the acquisition of personal information by others from the information itself; and the second is the stage of information processing, that is the stage of information processing after the completion of information collection. Focusing on the two stages of information circulation, I believe that the content of personal information personality right can be summarized as follows: First, the right of informed consent enjoyed by personal information in the stage of collection. That is to say, the user of information collection must obtain digitization of the information subject to collect and process its information, and Iization is out of the real will of the user, not forced consent under the obvious unequal status of the two parties. For example, for many applications on people's mobile phones, users must authorize operators to access the mobile phone address book, mobile phone album, and other permissions in order to obtain effective services. However, some access permissions are obviously not necessary for providing such services, and excessive collection of users' personal information exists. Personal information is in the acquisition phase, therefore, must obtain information, express or implied consent, this point is not only reflected in the information control people when collecting users' personal information must be in a reasonable way comprehensive, clear let me know the scope of information collection, the purpose and content will be processed, and information collection should follow the principle of minimization principle and the necessity. Any collection and use of information that goes beyond reasonable limits and beyond what is socially necessary to tolerate requires a re-authorization of the information itself. That is to say, if the information collection and processing company conducts operations beyond the scope of the initial authorization of the information subject on the user's personal information collected, it must obtain Iization of the information subject again (i.e., Iization of secondary utilization), otherwise it will constitute the violation of the informed consent right of the information subject. Second, the inquiry right of information subject to its information processing process. The existence of access right is of great significance for the information subject to realize its effective control over its own information. This right endows the information subject with the right to control the processing state of their personal information in real time, so as to effectively balance the unequal status between the information subject and the information controller and reduce the burden of proof of the information subject in the process of proof. In the judicial judgment of personal information protection in China, there are countless cases in which the plaintiff fails to provide sufficient evidence, although some scholars believe that special cases can be applied.

The burden of proof rule is used to coordinate the relationship between the information subject and the information collector, but I think that giving the information subject the right to query its information processing process is more conducive to the protection of personal information. No matter the burden of proof is inverted or reduced, this special burden of proof rule can only play a role in the process of litigation. For the right subject of personal information, it always belongs to the result of infringement in the process of litigation relief. it not only have exposed relief. Moreover, the right of access to personal information can make the information subject show real-time supervision and information collection and processing behavior before the infringement occurs, which is a preventive behavior in the nature of relief. Compared with the relief effect achieved by the special burden of proof rule, the personal information access right is obviously more advantageous. Third, the information subject has a series of intervening rights to object to the information controller's processing and utilization activities. The power can be viewed as the right of the above query subsequent power, found in information subject by querying the handling and use of their personal information conditions do not conform to the prior agreement, or harm the interests of my possibility, information main body in the process of information processing and utilization of information acquisition for disposal, seeking the relief to protect its own information. For example, if the information controller is found to have shared the collected personal information with a third party without authorization, the information controller may be required to stop processing and using his personal information and bear the corresponding tort liability. If the information controller is found to have disclosed wrong personal information, the information subject has the right to request correction or modification of the wrong information, or even withdrawal or deletion of the information that distorts the true image of the information.

#### 3.3.2. Property Interests

With the rapid development and widespread application of Internet information technology, personal information has been collected on a large scale and used in various commercial activities and social management activities, and its use value is particularly prominent. Under the function of market economy, the use of personal information can be reflected as a kind of property value and gradually become the wealth of citizens in the information society. The property interests of personal information can be reflected in the following two rights: first, the right to use information. This kind of information utilization has two meanings: the first layer can be expressed as the information subject's use of his personal information to meet his own needs according to his will. For example, information subjects voluntarily provide their personal information in order to obtain certain economic benefits or exchange for certain services. The second layer can be expressed as permission or restriction of information utilization other than information itself. For example, information subjects have the right to authorize others or forbid others to collect and process their personal information and have the right to require information collectors to use their information in a legitimate way within a reasonable range. Second, information usufruct. The biggest difference between the right to personal information and the right to privacy is that the information subject enjoys the right to profit from the use of his personal information, which is also the most prominent feature of the property right of personal information. It is worth noting that this right of earnings is not only expressed as the use of personal information to obtain direct economic benefits, but also can be expressed as the use of personal information in exchange for some social evaluation or service. Comparison in life.

It is common for job seekers to actively disclose their basic identity information, educational background, work experience, etc., in order to gain positive evaluation of the interviewer and ultimately succeed in the job search. Phone number and location are disclosed when using mobile ordering software to get food delivery service.

## 4. Discussion

In the current information society, people are increasingly aware of the importance of personal information, which has set off a tide of legislative protection of personal information in the world. The majority of domestic researchers believe that our country should develop a specific personal information protection law as quickly as possible, but this article acknowledges that due to the complexity of the personal information itself, the future of personal information protection law must also provide a framework of general provisions; for the regulation of personal information in the circulation of each hyperlink is still relevant, specific legal rules must be established accordingly. In addition, the protection of personal information can not only rely on upper-level legislation, but also need the active participation and cooperation of relevant regulatory departments, people engaged in various industries, and citizens. For the purposes of this article, we will mainly study the legal complications related to the right of personal information, describing the problems associated with personal information protection, such as how to carry out by the competent authority of the market regulation, how practitioners in each field of information security compliance, personal information in the process of circulation of different stages, etc. It may involve the knowledge principles of science and technology law, administrative law, information law, and other disciplines. In view of the limited academic ability of this article, the consideration of the above problems is not mature. I believe that in the subsequent research of scholars, these problems will be properly solved, so as to better grasp the balance between personal information protection and utilization and promote the sustainable development of China's digital economy.

## 5. Suggestion for Personal Information and Privacy Security Protection Measures

In this article, the four ways to protect personal information are proposed as:

### 5.1. Strengthen Industry Self-Discipline and Realize Self-Protection of Personal Information

The arrival of big data brings new challenges to personal information security. In recent years, countries all over the world have formulated relevant laws and policies to protect the privacy of individuals and ensure the security of personal information and privacy from disclosure. National laws and regulations is not perfect; however, China's laws and regulations, in particular, are too scattered. Legislation lags behind, disclosure of privacy can not be timely and effective punishment, which has become a prominent problem in the current social development. In order to strengthen industry self-discipline, industry standards are formulated according to the characteristics of the industry itself. Industry members should be encouraged to consciously abide by the rules and regulations for the protection of personal information, a sound industry internal management system and basic operating procedures should be established, and an initiative must be taken to accept the work guidance of public security organs and network supervision departments. Data collectors are guided to reasonably collect user information under the legal framework. The state and the industry shall establish special inspection and supervision mechanisms, advocate punishment and accountability systems, cultivate the moral quality of the industry personnel, form a good sense of social responsibility, strengthen the awareness of abiding by the law, and strictly regulate the collection and use of all kinds of data in the flow of information—clear personal information.

The qualifications of the collection and collection channels should be legal, and the purpose of using information should be informed to the holder of personal information. In the process of information storage, anonymous processing should be carried out so that the information subject cannot be identified, and transparency of the process of data transfer and circulation should be strengthened.

### 5.2. Improve Citizens' Awareness of Personal Information Protection

To protect personal information security, we can not only rely on the establishment and improvement of laws and regulations, strengthen industry self-discipline and improve the internal rules and regulations of enterprises, but also need to improve the awareness of personal information protection and protect their information security from the root. To develop good Internet habits, ambiguous websites should not be browsed or used. When using mobile devices such as mobile phones, Settings must be checked first and personal information must be protected. Therefore, from the national level, we can promote the protection of personal privacy in the media. We should strengthen the publicity of information security awareness, issue personal information security literature and thoroughly implement it, hold popular science lectures regularly, and release citizens' information security knowledge by using some network platforms. The government should include the protection of personal information into the protection and standardization of national strategic resources.

### 5.3. Establishing and Improving Laws and Regulations

The era of big data network increases the risk of personal information security to a large extent and makes it easier to leak personal privacy. Therefore, it is urgent to establish a set of perfect and operable personal information protection system; introduce “personal Information Protection Law” and “Privacy Law” as soon as possible; and make up for the legislative gap of personal privacy protection in our country. In the legal regulations, the following aspects of personal rights and obligations are mainly concerned. First, the obligation of clear disclosure. In China, citizens have weak awareness of personal information security, and enterprises or organizations should clearly inform information providers of the right to know and control when collecting personal information. Second, the way and purpose of use should be clarified. Information collectors and users should specify the purpose, storage location, scope, and period of use of collected personal data in detail. According to the policy requirements, personal information providers have the right to delete and modify, and excessive collection is not allowed. Again, pay attention to personality right, that shall not be arbitrarily filming, recording, leak, tracking the private activities of others, not for himself agreed to open, without authorization, buying and selling private information, such as personal privacy being invaded and take corresponding legal measures to stop, for mental damage to apologize restorable, information and economic compensation. In addition to bearing civil liability for the property loss of the victim, serious and harmful acts should be included in the category of criminal crime. Government supervision should be strengthened, a set of security assessment system must be established and implemented under the legal framework, and enterprises and individuals should be guided to strengthen the collection and management of private information. In addition, the accountability mechanism and punishment for the disclosure of individuals should be strengthened and foreign advanced management methods and laws and regulations should be learned to restrain the illegal behavior of enterprises or organizations.

### 5.4. Strengthen the Research on Personal Information Protection Technology in the Big Data Environment

At present, countries in the world take certain technologies to protect personal privacy from different perspectives, such as data encryption technology, data anonymization technology, data fuzzy technology, data interference technology, and differential privacy protection technology, to improve the efficiency of personal information.

## Figures and Tables

**Figure 1:** The relationship between big data and personal information and privacy.

**Table 1:** The legislative status of personal information right protection.

Region	Related legislation	Remark
European Union	Data Protection Directive, 1995	The general data protection regulations were further revised in 2014 and 2016, with the latest version coming into force in May 2018. To date, it is the latest and most comprehensive legal document on personal data protection in the international community.
	Directive No.95/46/EC/ of the European Parliament and of the Council on entry protection relating to the processing of entry data and the free circulation of such data, 1995	
	European Union Privacy Directive, 1998	
	Privacy and Electronic Communications Directive 2002	
	European Union Data Retention Directive, 2006	
	Draft No.2012/72 and 73 on the protection of individuals in relation to the processing of personal data and the free flow of such data, 2012	

	General data protection ordinance, 2012	
European commission	The 1981 convention on the protection of individuals in the automated processing of personal data was amended, 1999	
	Additional agreement on regulatory authorities and cross-border data flows to the convention on personal protection in the automated processing of personal data, 2001	
	Convention on personal protection in the processing of personal data, 2012	

Germany	The German state of Hesse enacted the Data Law of Hesse, the world's first specialized personal data protection law, 1970	The Federal Data Protection Act of 1977 stipulates that only with the consent of the parties concerned can personal data be collected, processed, and used, and the data parties have the right to know, correct, delete, and screen.
	Germany enacted a national Federal Data Protection Act, 1977	

Sweden	Swedish Data Act 1973	The world's first national personal data protection law
	Personal Data Act 1998 (supersedes the former)	

France	Information, Records and Freedom Act, 1978	

Britain	UK Data Protection Act, 1984	

Australia	The Privacy Act 1988 was passed in November 2012 and the Privacy Act Amendment Act came into force in March 2014	

Japan	Personal Information Protection Act, 1988	
	Law on the protection of personal data of administrative bodies in relation to computer processing, 1990	
	Personal Information Protection Act, 2003	

Malaysia	The Personal Data Protection Law was passed in 2010 and came into force on November 15, 2013	

America	The Fair Credit Reporting Act, 1970	
	Bank Secrecy Act, 1970	
	Fair Information General Rules, 1973	
	Privacy Act, 1974	
	Financial Privacy Act, 1978	
	Family Educational Rights and Privacy Act, 1978	
	Privacy Protection Act, 1980	
	Electronic Communications Secrecy Act, 1986	
	Federal Electronic Communications Privacy Protection Act, 1986	
	Computer Comparison and Privacy Protection Act, 1988	
	Telemarketing Consumer Protection Act, 1991	
	Consumer Credit Reporting Act, 1996	
	Children's Online Privacy Protection Act, 1998	
	National Cybersecurity and Critical Infrastructure Protection Law, 2002	
	Consumer Information Privacy Act, 2010	
	Internet Privacy Protection Act, 2012	
	Federal Privacy Act, 2014	
	California Online Privacy Protection Act, 2014	
	Privacy Shield Agreement, 2016	

Netherlands	Data Registration Act 1988; Personal Data Protection Act, 1999 (supersedes the former)	The Personal Data Protection Law of The Netherlands enacted in 1999 stipulates the following principles for government agencies to collect personal information: Personal data processing shall be carried out in accordance with the law and in a reasonable and appropriate manner; the collection of personal data must be accurate, authentic, and legitimate; the data subject has made an explicit consent to its own data processing; the processing of personal data should not exceed the scope of the data acquisition purpose; after the purpose of collection and processing of personal data is realized, the personal data shall not continue to be stored in the form of data subject being identified.

New Zealand	Privacy Act, 1993	There are 12 information privacy principles: The purpose of collecting individual information is legal; personal information comes from the person himself; rules for collecting information from the person; storage and security of personal information; get entry information; modify the input information; review of alignment and accuracy before use; the agency shall not hold personal information for longer than necessary; restrict the use of incoming information; restrictions on the disclosure of personal information; unique identification marks, etc.

OECD	Guidelines on privacy protection and cross-border flow of personal data, 1980	

United Nations General Assembly	Guidelines on specification of personal data documents for computer processing, 1990	

APEC	APEC Privacy Framework, 2004	

Taiwan, China	Computer Processing of Personal Data Protection Act, 1995	It regulates schools, hospitals, telecommunications, finance, and insurance.
	Personal Data Protection Act, 2012	The scope of use is extended to all industries. According to article 6, it classifies sensitive personal information based on whether it is related to individual core privacy, including “personal INFORMATION related to medical treatment, gene, sexual life, health examination, and criminal record.”

Hong Kong, China	Personal Data (Privacy) Ordinance, 1996. The Personal Data (Privacy) (Amendment) Ordinance was enacted in June, 2012	

## Data Availability

The experimental data of this study are available from the corresponding author upon request.
